# Validation of a 4-item child perception questionnaire in Australian children

**DOI:** 10.1371/journal.pone.0239449

**Published:** 2020-09-22

**Authors:** Xiangqun Ju, Pedro Henrique Ribeiro Santiago, Loc Do, Lisa Jamieson

**Affiliations:** Australian Research Centre for Population Oral Health, Adelaide Dental School, The University of Adelaide, Adelaide, SA, Australia; Centre Hospitalier Regional Universitaire de Tours, FRANCE

## Abstract

**Objective:**

To develop and validate a 4-item child oral health-related quality of life (OHRQoL) instrument that might be more amenable for uptake in large scale, multifaceted surveys of children’s health and wellbeing than current, longer-form child OHRQoL instruments.

**Methods:**

Data were obtained from a study of the South Australian School Dental Service population designed to investigate OHRQoL among school children aged 8–13 years in 2002–2003. The Child Perception Questionnaire (CPQ_8-10_ and CPQ_11-14_) was utilised, which comprises 25 & 37 items representing four conceptual domains: oral symptoms, functional limitations, emotional wellbeing and social wellbeing. Initially, the psychometric properties of the short form 8-item CPQ were tested in both age groups using Confirmatory Factor Analysis. The rationale was that, if the 8-item CPQ_8-10_ and CPQ_11-14_ did not display good psychometric properties, there was no reason to proceed with further shortening into 4-item versions. Following a good fit of the 8-item CPQ, items with higher factor loadings in each domain were maintained and tested in the development of a 4-item CPQ. Exploratory Factor Analysis was conducted to determine dimensionality, followed by tests for reliability and validity. Model fits were assessed using Root Mean Square Error of Approximation (RMSEA), Comparative Fit Index (CFI) and Standardized Root Mean Square Residual (SRMR).

**Results:**

There were 308 children aged 8–10 years who completed CPQ_8-10_ and 461 children aged 11–13 years who completed CPQ_11-14_. For the short-form 8-item instrument, satisfactory goodness of fit was demonstrated for the two age groups, with acceptable thresholds for RMSEA, CFI, and SRMR. The four items with the highest factor loading in each domain were the same for the 8-item CPQ_8-10_ and CPQ_11-14._ and these items were selected to comprise the 4-item CPQ_8-10_ and CPQ_11-14._ The 4-item short form displayed good criterion validity, with expected score patterns found in the majority of the known groups evaluated.

**Conclusions:**

We developed short-form 4-item CPQ_8-10_ and CPQ_11-14_ instruments that were tested in a large convenience sample of South Australian school children. The instruments demonstrated acceptable reliability and validity. Implications for practice are discussed.

## Intrduction

Oral health is an important component of overall health and wellbeing, and is a fundamental human right [1]. Poor oral health has a substantial impact on a child’s overall wellbeing and engagement, frequently necessitating expensive treatment under a general anaesthetic and resulting in substantial time away from school [2]. It impacts on academic performance, on ability to make meaningful social engagements and to thrive in the school environment over the long term [3, 4]. In Australia, dental conditions are one of the highest causes of acute preventable hospital admissions for children [5]. Undesirable dental aesthetics in childhood contributes to poor social and emotional wellbeing through decreased self-confidence, embarrasment and avoidance of social interactions [6]. Poor childhood oral health also leads to substantial financial burdens being placed on the individual, community and health-care system [7]. Lack of access to service providers is frequently cited as a reason for poor child oral health, together with specific behavioural risk factors and social determinants [8]. In Australia’s 2012–14 National Child Oral Health Survey, 42 percent of children aged 5 to 10 years had experience of dental disease [9]. Including an assessment of oral health-related child wellbeing is a crucial, but frequently overlooked, component in examining risk factors for failure to flourish during the formative years of a child’s academic life. This, in turn, has long term impacts on social productivity and social capital [10].

For many decades in Australia, dental service provision for children was without cost (or required small co-payments), and occurred onsite in school-based dental clinics. This is regrettably no longer the case in most jurisdictions. Many school children now receive dental care privately, through the Child Dental Benefits scheme, or through specialist paediatric dentists. In many instances, untreated dental disease may first be observed in the classroom (child complaining of toothache, irritability, not concentrating in class, not wanting to engage socially). Because of these immediate impacts, and the consequence of poor oral health in long term educational achievements, it would be helpful to have a tool that assesses child wellbeing and engagement as it relates to oral health that could be readily utilised within administrative data collections within education and other government departments, as well as in large national and population based surveys.

Several instruments have been developed to assess the contribution of poor oral health to overall child wellbeing and engagement. The most internationally validated of these is the Child Perception Questionnaire for use among children aged 8 to 10 years (CPQ_8-10_) and children aged 11 to 14 years (CPQ_11-14_) [11, 12]. The CPQ_11-14_ comprised 37 items that captured four fundamental domains relating to child oral health-related quality of life: (1) oral symptoms; (2) functional limitations; (3) emotional wellbeing and; (4) social wellbeing. In the initial CPQ_11-14_ validation, a large item pool was developed by interviewing parents and health professionals who treated children with oral and orofacial disorders. Children aged 11 to 14 years then appraised all items and indicated the ones which best reflected their most frequent and bothersome oral health-related problems. For instance, items such as “Avoided smiling when around other children” were retained, while items such as “Difficulty doing homework” were excluded. In the end, 37 items were selected to compose the initial version of the CPQ_11-14_. The 37-item CPQ_11-14_ displayed excellent internal consistency (α = 0.91) and test-retest reliability (ICC = 0.90) [11] and was validated in different contexts, including in a large representative sample in Australia [13].

Despite its good psychometric properties, application of the 37-item CPQ_11-14_ in both clinical settings and health research is limited due to its length and response burden [14]. Response burden leads to low response rates, increased item response missingness and is particularly problematic for specific demographic groups, for instance, children [15]. For this reason, subsequent research efforts focused on developing shortened CPQ versions such as the 25-item CPQ_8-10_ [12], the 16-item CPQ_11-14_ and 8-item CPQ_11-14_ [16]. These short forms displayed good psychometric properties, including excellent criterion validity. For example, mean scores for the 16-item CPQ_11-14_ and 8-item CPQ_11-14_ were higher for children with 10 or more decayed tooth surfaces compared to those with fewer than 10 decayed tooth surfaces. There was high agreement (Spearman’s ρ from 0.87 to 0.95) between the CPQ_11-14_ short-forms and 37-item CPQ_11-14_ scores [16]. Recently, investigators in an international collaborative study re-evaluated the validity of the 16-item CPQ_11-14_, this time using a large sample of children (n = 5,804) from countries including Australia, New Zealand, Brunei, Cambodia, Hong Kong, Malaysia, Thailand, England, Germany, Mexico and Germany. Thomson et al. [17] concluded that the CPQ_11-14_ performed well, on the whole, across most countries with psychometric properties that were mostly consistent. One concern with the 8- and 16-item CPQ_11-14_, however, was the decreased reliability compared to the excellent reliability found in the original 37-item CPQ_11-14_ (α = 0.91, ICC = 0.90) [16]. Since reliability is a function of questionnaire length and trait variance, it is widely documented that shortening a questionnaire frequently decreases its reliability [18]. Jokovic et al. [16] discussed how, in relation to the 8- and 16-item CPQ_11-14_, the short-forms’ reliability (ranging from 0.71 to 0.83) still exceeded standards for group-level comparison but cautioned against the use of short forms in small cross-sectional studies, particularly when the samples show low OHRQoL variations. The same holds for individual-level assessments since they require that reliability coefficients are at least 0.90.

In summary, despite successful development of the 8- and 16-item CPQ_11-14_ [16] and the 25-item CPQ_8-10_ [12], there has been no uptake of these short forms in many government-funded surveys of school children in part because, for logistical, pragmatic and financial reasons, the instrument is still considered to be too long. Because a shorter form could have many potential applications, for example, inclusion in government surveys in Australia such as the Longitudinal Study of Australian Children and Longitudinal Surveys of Australian Youth, our aims were to develop and test the validity of 4-item CPQ_8-10_ and CPQ_11-14_ instruments. Our hypothesess were that: (1) 4-item versions of the CPQ_8-10_ and CPQ_11-14_ would have adequate psychometric properties and; (2) the 4-items measure a single overall dimension of children's OHRQoL.

## Methods

### Sample

Data were obtained from a study of the South Australian School Dental Service population designed to investigate OHRQoL among school children aged 8–13 years in 2002–2003 [13].

Children and their parents were approached with a package containing an information letter, a consent form and questionnaires. Parents provided signed informed consent. A total of 1,401 children were sampled, with 842 parent/child pairs responding with completed questionnaires. Data for this analysis comprises 308 children aged 8–10 years who completed CPQ_8-10_ and 461 children aged 11–13 years who completed CPQ_11-14_. Ethical approval was granted by the Human Research Ethics Committee of the University of Adelaide.

### The child perception questionnaire (CPQ)

The CPQ is designed to measure children’s OHRQoL. The short form CPQ_8-10_ from the 25-item CPQ_8-10_ and 37-item CPQ_11-14_ [13] comprises 8 items and represents 4 conceptual domains: oral symptoms (OS_1_: ‘Pain’ and OS_2_: ‘Food stuck or caught’), functional limitation (FL_1_: ‘Difficulty biting or chewing firm food’ and FL_2_: ‘Taken longer than others to eat a meal‘), emotional wellbeing (EW_1_: ‘Been upset because of problems with your teeth, lips, mouth or jaws’ and EW_2_: ‘Been irritable or frustrated because of problems with your teeth, lips, mouth or jaws’) and social wellbeing (SW_1_: ‘Missed school because of problems with your teeth, lips, mouth or jaws’ and SW_2_: ‘Not wanted to talk to other children because of problems with your teeth, lips, mouth or jaws’) (**Table 1**). Each item is ranked on 5-point Likert scale ranging from 1 to 5 (1 = Never, 2 = Once or twice, 3 = Sometimes, 4 = Often, and 5 = Very often). Scores were re-coded: 1 to 0, 2 to 1, 3 to 2, 4 to 3, and 5 to 4. Summary scores ranged from 0–16, after re-coding, with higher total scores indicating worse child OHQoL.

**Table 1:** The 8-item child perception questionnaire (CPQ_8-10_ and CPQ_11-14_).

	Items	CPQ_8-10_	CPQ_11-14_
**CPQ questions**	During the last 3 months, how often have you had…‥		
Oral symptoms (OS)	**OS**_**1**_**: Pain**	Pain in teeth or mouth	Pain in teeth, lips, mouth or jaws
	OS_2_: Food stuck or caught	Food stuck in your teeth	Food caught in or between your teeth
Functional limitation (FL)	**FL**_**1**_**: Difficulty biting or chewing firm foods**	Had a hard time to bite or chew food like apples, carrots, nuts or steak	Difficult to bite or chew food like apples, carrots, nut, or steak
	FL_2_: Taken longer than others to eat a meal	Needed longer time than others to eat your meal	Taken longer than others to eat a meal
Emotional wellbeing (EW)	**EW**_**1**_**: Been upset**	Been upset because of your teeth or mouth	Been upset
	EW_2_: Been irritable or frustrated	Felt frustrated because of your teeth or mouth	Felt irritable or frustrated
Social wellbeing (SW)	SW_1_: Missed school	Missed school because of pain, appointments, or surgery	Missed school because of pain, appointments, or surgery
	**SW**_**2**_**: Not wanted to talk to other children**	Not wanted to talk to other children because of your teeth or mouth	Not wanted to talk to other children
**Response options**		Never/Once or twice/ Sometimes/Often/Very often	Never/Once or twice/ Sometimes/Often/Very often

The items which composed the 4-item CPQ_8-10_ and CPQ_11-14_ are highlighted in bold.

### Criterion validity

Covariates used in the analysis of criterion validity included sociodemographic, dental health-related, self-rated oral health, and dental disease-related characteristics. Self-rated oral health was measured with the question “How would you rate your dental health?”, with response options (Very good/Good/OK/Poor) for children aged 8 to 10 and response options (Excellent/Very good/Good/Fair/Poor) for children aged 11 to 13. The sociodemographic characteristics included children’s sex (boy vs girl), parent answering the survey’s highest education level (High school or less, Trade to Diploma or Tertiary) and; annual household income (<AUS$40K, AUS$40-60K or >AUS$60K: ‘1AUS$ = 0.7US$’). The dental health-related behaviours included: frequency of tooth brushing (≥2/day vs <2/day), consumption of soft drinks (twice a day or more vs once a day or less), and consumption of sweet drinks (twice a day or more vs once a day or less). The response options for child’s self-rated oral health included ‘excellent/very good’ vs ‘good/fair/poor. Dental caries experience was collected from each child’s School Dental Service clinic records: decayed (d/D), missing (m/M) and filled (f/F) teeth. Dental caries experience (% dmft/DMFT≥1) and untreated decay (% dt/DT≥1) were categorised as ‘Yes vs No’.

### Statistical analysis

Data was stratified into two age groups: children aged 8–10 years and children aged 11–13 years. To evaluate the validity of 4-item versions of the CPQ_8-10_ and CPQ_11-14_ we conducted two steps. The first step was to investigate the validity of the 8-item CPQ_8-10_ and CPQ_11-14_ using Confirmatory Factor Analysis (CFA). In both instruments, the factorial structure evaluated was the 4-factor model (i.e. oral symptoms, functional limitation, emotional wellbeing and social wellbeing) with 2 items per factor (**Table 1**). Although the 8-item version displayed good psychometric properties in other contexts, such as New Zealand [14], it is still necessary to ensure that it has good psychometric properties for children in the current study. The rationale is that, if the 8-item CPQ_8-10_ and CPQ_11-14_ do not display good psychometric properties for the children in question, there is no reason to proceed with further shortening into 4-item versions.

The CFA models were estimated with maximum likelihood [19]. Model fit was assessed using the chi-square test statistic (χ_2_), Comparative Fit Index (CFI), Root Mean Square Error of Approximation (RMSEA) and Standardized Root Mean Square Residual (SRMR). Model fit was considered acceptable when CFI>0.96, RMSEA<0.8 and SRMR <0.08 [20–23]. When acceptable fit of the 8-item version was established, the four items with the highest factor loading on each domain was selected to comprise the 4-item CPQ_8-10_ and 4-item CPQ_11-14_. The factor loading indicates how much item responses were influenced by the underlying construct they intend to measure (rather than influenced by measurement error) [24]. Hence, the CPQ_8-10_ and CPQ_11-14_ items with highest factor loadings were the ones most influenced by (and, consequently, which better measured) their respective OHRQoL domains (i.e. oral symptoms, functional limitation, emotional wellbeing and social wellbeing).

After choosing the 4 items with the highest factor loading, the second step was to test the dimensionality of the 4-item CPQ_8-10_ and CPQ_11-14_ instruments using Exploratory Factor Analysis (EFA). Considering that 4-item CPQ_8-10_ and CPQ_11-14_ versions have never been evaluated, we did not have any prior information on possible factorial structures. In this case, when factorial structures are unknown, EFA should be preferred over CFA [25]. The quality of the factor analysis models was assessed using the Kaiser-Meyer-Olkin (KMO) test and Bartlett´s test for sphericity. The KMO test measures the degree of multi-collinearity (based on partial correlations) between the included items, varies between 0 and 1 and should be greater than 0.5–0.6. Bartlett’s test is a measure of the probability that the initial correlation matrix is an identity matrix and should be under 0.05. Factor retention was evaluated with Scree Plots, and remained satisfactory if their primary factor loading was more than 0.40 [26]. Finally, Cronbach’s α and corrected item total correlations (CITCs) were used to assess the internal consistency of the instruments. A Cronbach’s α coefficient of 0.70 or higher is considered satisfactory [27, 28]. A CITC value lower than 0.30 indicates that an item displays poor internal consistency with the other items and should be excluded.

Criterion validity of the 4-item CPQ_8-10_ and CPQ_11-14_ instruments was tested by examining known-groups comparisons [29]. That is, the extent to which groups expected to display worse OHRQoL (e.g. less educated, higher dmft, worse self-rated oral health) had higher scores (indicates worse OHRQoL) in the 4-item CPQ_8-10_ and CPQ_11-14_. The 4-item CPQ_8-10_ and CPQ_11-14_ instruments were thus stratified by socio-demographic, dental behaviours, self-rated oral health and dental disease-related characteristics. All data were analysed using SAS statistical software (SAS 9.4, SAS Institute Inc., Cary, NC, USA).

## Results

The CFA results of the 8-item CPQ_8-10_ and CPQ_11-14_ are presented in **Table 2**. Satisfactory goodness of fit was demonstrated with acceptable thresholds for RMSEA, CFI and SRMR. In addition, the four items with highest factor loading were the same for the 8-item CPQ_8-10_ and the CPQ_11-14_ (OS_1_, FL_1_, EW_1_ and SW_2_) (see **Table 1**: items in bold pertain). We selected these 4 items and proceeded to evaluate the validity and reliability of the 4-item CPQ_8-10_ and CPQ_11-14._

**Table 2:** Confirmatory factor analysis of the 8-item CPQ_8-10_ and CPQ_11-14_.

Items	Aged 8–10 years (n = 308)				Aged 11–13 years (n = 461)			
	CPQ_8-10_					CPQ_11-14_		
	Mean (SD)	Median (IQR)	Factor loading	95% CI	Mean (SD)	Median (IQR)	Factor loading	95% CI
**OS**_**1**_	0.70 (0.85)	0 (0–1)	**0.507**	**0.36–0.66**	0.78 (0.87)	1 (0–1)	**0.670**	**0.56–0.66**
OS_2_	1.55 (1.00)	1 (1–2)	0.358	0.23–0.49	1.54 (1.03)	1 (1–2)	0.419	0.32–0.52
**FL**_**1**_	0.62 (0.89)	0 (0–1)	**0.531**	**0.41–0.65**	0.58 (0.92)	0 (0–1)	**0.782**	**0.70–0.86**
FL_2_	0.42 (0.79)	0 (0–1)	0.530	0.41–0.65	0.49 (0.95)	0 (0–1)	0.582	0.50–0.66
**EW**_**1**_	0.38 (0.76)	0 (0–1)	**0.732**	**0.64–0.83**	0.19 (0.54)	0 (0–0)	**0.762**	**0.71–0.82**
EW_2_	0.44 (0.82)	0 (0–1)	0.714	0.62–0.81	0.35 (0.70)	0 (0–0)	0.738	0.68–0.79
SW_1_	0.20 (0.50)	0 (0–0)	0.638	0.46–0.83	0.19 (0.55)	0 (0–0)	0.521	0.44–0.61
**SW**_**2**_	0.09 (0.38)	0 (0–0)	**0.639**	**0.46–0.82**	0.22 (0.61)	0 (0–0)	**0.602**	**0.52–0.69**
**Chi-square**			44.34				22.66	
**DF**			14				14	
**P-value**			0.009				<0.001	
**RMSEA**			0.053				0.069	
**CFI**			0.970				0.967	
**SRMR**			0.033				0.035	

**DF**: degrees of freedom; **RMSEA**: root mean square error of approximation; **CFI**: Bentler comparative fit index; **SRMR**: Standardized root mean square residual. The highest factor loadings for each factor are displayed in bold.

CI: confidence interval

IQR: Interquartile range (being equal to the difference between 75th and 25th percentiles)

**Table 3** shows the EFA results of the 4-item CPQ_8-10_ and CPQ_11-14_. The KMO values were over 0.6 and Bartlett’s tests were under 0.05 in both the 4-item CPQ_8-10_ and CPQ_11-14_ instruments. This supports the factorability of correlation matrices and demonstrates the suitability of the data for the factor analysis. The EFA results indicate that the eigenvalues of the first factors were substantially higher than the eigenvalues of the three other factors. These results can be seen in the Scree Plots (**Fig 1**).

**Fig 1:** Scree plots of the 4-item CPQ_8-10_ and CPQ_11-13_.

**Table 3:** 4-item CPQ descriptive, reliability and factor analysis.

Items	Factor loadings	^a^CITC
**Aged 8–10 years**		
OS_1_	0.77	0.47
FL_1_	0.68	0.33
EW_1_	0.72	0.37
SW_2_	0.41	0.21
Kaiser-Meyer-Olkin’s test: 0.60, range: 0.57–0.62		
Bartlett’s test of sphericity: 0.0022		
Eigenvalues: F1 = 1.73; F2 = 0.99; F3 = 0.74; F4 = 0.54		
Cumulative variance explained (%): F1 = 0.43; F2 = 0.68; F3 = 0.87; F4 = 1.00		
Cronbach standardized alpha (α): 0.57		
**Aged 11–13 years**		
OS_1_	0.63	0.38
FL_1_	0.74	0.49
EW_1_	0.76	0.50
SW_2_	0.72	0.45
Kaiser-Meyer-Olkin’s test: 0.63, range: 0.61–0.66		
Bartlett’s test of sphericity: <0.0001		
Eigenvalues: F1 = 2.03; F2 = 0.96; F3 = 0.55; F4 = 0.45		
Cumulative variance explained (%): F1 = 0.51; F2 = 0.75; F3 = 0.87; F4 = 1.00		
Cronbach standardized alpha (α): 0.68		

^a^**CITC**: Corrected Item-Total Correlation

Furthermore, the eigenvalues of the second factor were smaller than 1 for both the CPQ_8-10_ (Λ = 0.99) and CPQ_11-14_ (Λ = 0.99). In the absence of measurement error, the second, third and fourth factor would explain less variance of the item responses than a single item, which is unacceptable. Hence, the evaluation of the Scree plots indicated that one factor should be retained. That is, the 4-item CPQ_8-10_ and CPQ_11-13_ are unidimensional instruments since they measure a single overall OHRQoL factor. Furthermore, factor loading values were nearly or higher than 0.7 for all items, with the exception of item SW_2_ (λ = 0.41), indicating that the factor substantially explained the variance from item responses. Furthermore, factor loading values were higher than 0.40 for all items, indicating that the factor substantially explained the variance from item responses.

Cronbach’s standardized alpha was nearly 0.7 in the 11–13 years group (0.68), which appeared to have good internal consistency; but less than 0.7 in the younger group (0.56). The total item correlation values were more than 0.3, except for SW_2_ (0.2) in the younger age group, which indicated that each item correlates well with the scale overall. In addition, the correlation between each item (representing each domain) of the 4-item CPQ, and each domain and total score of the 8- and 25-item CPQ_8-10_ and 31-item CPQ _11–14_ (see **Table 4)** indicated medium to strong correlations (ranging from 0.55 to 0.86) between each domain of the 4-item, and the 8- /25- /31-item CPQ. The exception was SW_2_ of the 4-item with the total 25/31-item CPQ (0.37 and 0.44, respectively).

**Table 4:** Correlation between the 4-item, 8- and 25/31-item CPQ _8–10_ and CPQ _11–1_.

		^a^ **The 8 item CPQ**_**8-10**_		^b^ **The 25-item CPQ**_**8-10**_	
	**The 4-item CPQ**_**8-10**_	Each domain	Total	Each domain	Total
Oral symptoms **(OS)**	Pain in teeth or mouth (**OS**_**1**_)	0.72	0.65	0.62	0.56
Functional limitation **(FL)**	Had a hard time to bite or chew food like apples, carrots, nuts or steak (**FL**_**1**_**)**	0.83	0.61	0.75	0.56
Emotional wellbeing **(EW)**	Been upset because of your teeth or mouth **(EW**_**1**_**)**	0.86	0.66	0.73	0.66
Social wellbeing **(SW)**	Not wanted to talk to other children because of your teeth or mouth **(SW**_**2**_**)**	0.78	0.44	0.67	0.37
	**Total scores**		0.52		0.66
		^c^ **The 8 item CPQ**_**11-14**_		^d^ **The 31-item CPQ**_**11-14**_	
	**The 4-item CPQ**_**11-13**_	Each domain	Total	Each domain	Total
Oral symptoms **(OS)**	Pain in teeth, lips, mouth or jaws **(OS**_**1**_**)**	0.76	0.65	0.64	0.55
Functional limitation **(FL)**	Difficult to bite or chew food like apples, carrots, nut, or steak **(FL**_**1**_**)**	0.85	0.72	0.74	0.61
Emotional wellbeing **(EW)**	Been upset because of your teeth or mouth **(EW**_**1**_**)**	0.85	0.64	0.73	0.70
Social wellbeing **(SW)**	Not wanted to talk to other children (**SW**_**2**_**)**	0.83	0.59	0.69	0.63
	**Total scores**		0.73		0.87

^a:^ 2 items for each domain

^b:^ 5 items for OS, FL and EW, and 10 items for SW;

^c:^ 2 items for each domain;

^d:^ 6 items for OS, 7 items for FL, 8 items for EW and 10 items for SW.

After establishment of the factorial structure, the next step was evaluation of the 4-item CPQ_8-10_ and CPQ_11-14_ criterion validity. **Tables 5 and 6**demonstrate the instrument scores stratified by related covariates. For those aged 8–10 years, higher scores were observed for either the total 4-item instrument and/or individual CPQ items among those with ‘Ok/Poor’ self-ratings of oral health, experience of dental caries, consumption of sweet drinks twice a day or more. For those aged 11–13 years, higher scores were observed for either the total 4-item CPQ instrument and/or individual CPQ items among those who rated their oral health as fair or poor, had experience of dental caries, consumed sweet drinks twice a day or more, had an annual household income of $40–60,000 Australian. In addition, 8-item CPQ_8-10_ and CPQ_11-14_ criterion validity was evaluated, and the same results were observed in most domains and total CPQ (see **Tables 7 and 8**).

**Table 5:** Mean (SE) scores for 4-item CPQ and individual items by sample characteristics among children aged 8–10 years.

		The child perception questionnaire (CPQ)				
		Oral symptoms	Functional limitation	Emotional wellbeing	Social wellbeing	CPQ
	N (%)	Mean (SE)	Mean (SE)	Mean (SE)	Mean (SE)	Mean (SE)
Total	308	**0.70 (0.05)**	**0.63 (0.05)**	**0.38 (0.04)**	**0.09 (0.02)**	**1.90 (0.11)**
**Sex**						
Boy	160 (52.0)	0.72 (0.07)	0.56 (0.07)	0.33 (0.06)	0.22 (0.04)	1.81 (0.16)
Girl	148 (48.1)	0.68 (0.07)	0.70 (0.07)	0.44 (0.06)	0.18 (0.04)	1.99 (0.16)
**Parent’s Education level**						
High school or less	141 (49.3)	**0.71 (0.04)**	0.54 (0.07)	0.40 (0.05)	0.09 (0.03)	1.77 (0.16)
Trade to diploma	63 (22.0)	0.65 (0.09)	0.70 (0.11)	0.26 (0.05)	0.13 (0.04)	**1.97 (0.24)**
Tertiary	82 (28.7)	**0.62 (0.03)**	0.68 (0.10)	0.26 (0.04)	0.04 (0.04)	1.74 (0.21)
**Household income**						
< ^a^AUS$ 40k	107 (39,5)	0.64 (0.08)	0.59 (0.09)	0.36 (0.06)	0.05 (0.03)	1.72 (0.18)
AUS$ 40-60k	76 (28.0)	0.72 (0.10)	0.67 (0.10)	0.36 (0.07)	0.15 (0.04)	1.89 (0.22)
>AUS$ 60k	88 (32.5)	0.63 (0.09)	0.59 (0.09)	0.25 (0.07)	0.06 (0.04)	1.67 (0.20)
**Soft drink daily**						
Twice a day or more	123 (42.9)	**0.78 (0.07)**	**0.68 (0.08)**	**0.42 (0.06)**	**0.11 (0.03)**	**2.06 (0.17)**
Once a day or less	164 (57.1)	**0.60 (0.04)**	**0.52 (0.04)**	**0.26 (0.03)**	**0.05 (0.02)**	**1.62 (0.11)**
**Sweet drink**						
Twice a day or more	93 (32.4)	**0.79 (0.06)**	**0.69 (0.06)**	0.33 (0.07)	0.07 (0.04)	**1.94 (0.11)**
Once a day or less	194 (67.6)	**0.63 (0.05)**	**0.56 (0.04)**	0.34 (0.05)	0.09 (0.03)	**1.70 (0.12)**
**Tooth brushing**						
<2/day	76 (27.1)	0.54 (0.10)	0.53 (0.10)	0.32 (0.08)	**0.12 (0.03)**	**1.88 (0.13)**
≥ 2/day	204 (72.9)	0.72 (0.06)	0.64 (0.06)	0.34 (0.05)	**0.07 (0.02)**	**1.55 (0.12)**
**dmft ≥1**						
Yes	133 (51.4)	**0.95 (0.07)**	0.60 (0.08)	0.39 (0.07)	**0.14 (0.02)**	**1.99 (0.12)**
No	126 (48.7)	**0.70 (0.06)**	0.68 (0.08)	0.42 (0.07)	**0.06 (0.03)**	**1.54 (0.11)**
**dt≥1**						
Yes	45 (18.2)	0.58 (0.13)	0.51 (0.13)	0.36 (0.11)	**0.15 (0.03)**	1.71 (0.31)
No	202 (81.8)	0.70 (0.06)	0.60 (0.06)	0.39 (0.05)	**0.06 (0.02)**	1.87 (0.14)
**Self-rate oral health**						
Ok/poor	116 (39.5)	**0.92 (0.06)**	**0.89 (0.06)**	**0.51 (0.06)**	0.07 (0.03)	**2.46 (0.18)**
Ex/Very good/good	178 (60.5)	**0.54 (0.06)**	**0.47 (0.06)**	**0.23 (0.05)**	0.07 (0.02)	**1.44 (0.14)**

Patterns where expected values (p<0.05) were found are displayed in bold. For example, it was expected that children with worse self-rated oral health would display higher CPQ scores, indicating worse OHRQoL;

^a^1AUS$ = 0.7US$

**Table 6:** Mean (SE) scores for 4-item CPQ and individual items by sample characteristics among children aged 11–13 years.

		The child perception questionnaire (CPQ)				
		Oral symptoms	Functional limitation	Emotional wellbeing	Social wellbeing	CPQ
	N (%)	Mean (SE)	Mean (SE)	Mean (SE)	Mean (SE)	Mean (SE)
Total	461	0.79 (0.04)	0.59 (0.04)	0.19 (0.03)	0.22 (0.03)	1.75 (0.10)
**Sex**						
Boy	232 (50.3)	0.84 (0.07)	0.62 (0.06)	0.17 (0.04)	0.21 (0.04)	1.84 (0.14)
Girl	229 (49.7)	0.73 (0.06)	0.56 (0.06)	0.22 (0.04)	0.15 (0.04)	1.65 (0.14)
**Parent’s Education level**						
High school or less	178 (40.6)	0.77 (0.07)	0.60 (0.07)	**0.25 (0.02)**	0.23 (0.05)	**1.78 (0.11)**
Trade to diploma	106 (24.2)	0.84 (0.09)	0.61 (0.09)	**0.15 (0.03)**	0.19 (0.06)	**1.74 (0.21)**
Tertiary	154 (35.2)	0.76 (0.07)	0.53 (0.08)	0.19 (0.04)	0.20 (0.05)	**1.60 (0.13)**
**Household income**						
< ^a^AUS$ 40k	165 (39.9)	0.75 (0.07)	0.60 (0.07)	0.23 (0.04)	**0.26 (0.03)**	**1.79 (0.14)**
AUS$ 40-60k	127 (30.7)	0.93 (0.08)	0.52 (0.08)	0.17 (0.05)	**0.14 (0.05)**	1.73 (0.19)
>AUS$ 60k	122 (29.5)	0.64 (0.08)	0.53 (0.08)	0.16 (0.05)	0.24 (0.06)	**1.49 (0.11)**
**Soft drink daily**						
Twice a day or more	189 (42.8)	**0.84 (0.03)**	**0.64 (0.05)**	**0.23 (0.03)**	0.23 (0.05)	**1.91 (0.14)**
Once a day or less	253 (57.2)	**0.74 (0.03)**	**0.50 (0.03)**	**0.17 (0.02)**	0.21 (0.04)	**1.61 (0.11)**
**Sweet drink daily**						
Twice a day or more	147 (33.3)	0.79 (0.08)	0.59 (0.08)	**0.23 (0.03)**	**0.31 (0.05)**	**1.85 (0.12)**
Once a day or less	295 (66.7)	0.78 (0.05)	0.58 (0.06)	**0.16 (0.02)**	**0.18 (0.03)**	**1.69 (0.08)**
**Tooth brushing**						
<2/day	145 (34.1)	**0.84 (0.06)**	0.57 (0.08)	0.15 (0.04)	**0.26 (0.03)**	1.71 (0.18)
≥ 2/day	280 (65.9)	**0.76 (0.04)**	0.60 (0.06)	0.18 (0.03)	**0.19 (0.02)**	1.70 (0.13)
**DMFT ≥1**						
Yes	101 (29.0)	**0.90 (0.08)**	**0.69 (0.09)**	**0.27 (0.05)**	**0.32 (0.06)**	**2.05 (0.20)**
No	247 (71.0)	**0.70 (0.03)**	**0.47 (0.05)**	**0.14 (0.03)**	**0.17 (0.04)**	**1.48 (0.14)**
**DT≥1**						
Yes	27 (7.2)	**0.96 (0.14)**	0.56 (0.18)	**0.28 (0.05)**	**0.28 (0.03)**	**1.96 (0.24)**
No	350 (92.8)	**0.76 (0.05)**	0.55 (0.05)	**0.17 (0.03)**	**0.23 (0.03)**	**1.66 (0.08)**
**Self-rate oral health**						
Fair/poor	39 (12.3)	**1.18 (0.14)**	**1.13 (0.14)**	**0.56 (0.08)**	**0.46 (0.10)**	**3.26 (0.31)**
Ex/Very good/good	278 (87.7)	**0.72 (0.05)**	**0.50 (0.05)**	**0.12 (0.03)**	**0.19 (0.04)**	**1.46 (0.11)**

Patterns where expected values (p<0.05) were found are displayed in bold. For example, it was expected that children with worse self-rated oral health would display higher CPQ scores, indicating worse OHRQ

^a^1AUS$ = 0.7US$

**Table 7:** Mean (SE) scores for 8-item CPQ and individual items by sample characteristics among children aged 8–10 years.

		The child perception questionnaire (CPQ)				
		Oral symptoms	Functional limitation	Emotional wellbeing	Social wellbeing	CPQ
	N (%)	Mean (SE)	Mean (SE)	Mean (SE)	Mean (SE)	Mean (SE)
Total	308	2.24 (0.08)	1.04 (0.09)	0.81 (0.08)	0.29 (0.04)	4.37 (0.22)
**Sex**						
Boy	160 (52.0)	2.24 (0.11)	0.91 (0.11)	0.72 (0.11)	0.32 (0.06)	4.19 (0.28)
Girl	148 (48.1)	2.24 (0.12)	1.17 (0.11)	0.92 (0.11)	0.26 (0.06)	4.56 (0.29)
**Parent’s Education level**						
High school or less	141 (49.3)	2.24 (0.12)	0.89 (0.11)	**0.89 (0.08)**	**0.24 (0.06)**	4.15 (0.28)
Trade to diploma	63 (22.0)	2.25 (0.18)	1.21 (0.17)	**0.60 (0.07)**	**0.46 (0.08)**	4.56 (0.42)
Tertiary	82 (28.7)	2.02 (0.16)	1.02 (0.15)	0.76 (0.10)	**0.19 (0.07)**	3.99 (0.37)
**Household income**						
< ^a^AUS$ 40k	107 (39,5)	2.13 (0.14)	0.97 (0.13)	0.78 (0.12)	0.17 (0.06)	4.07 (0.32)
AUS$ 40-60k	76 (28.0)	2.37 (0.16)	1.07 (0.15)	0.76 (0.14)	0.29 (0.07)	4.50 (0.38)
>AUS$ 60k	88 (32.5)	2.00 (0.15)	0.98 (0.14)	0.64 (0.13)	0.26 (0.06)	3.89 (0.35)
**Soft drink daily**						
Twice a day or more	123 (42.9)	**2.37 (0.16)**	1.07 (0.12)	**0.89 (0.08)**	**0.35 (0.05)**	**4.56 (0.28)**
Once a day or less	164 (57.1)	**2.01 (0.07)**	0.93 (0.09)	**0.60 (0.07)**	**0.20 (0.03)**	**3.65 (0.20)**
**Sweet drink**						
Twice a day or more	93 (32.4)	**2.35 (0.10)**	0.99 (0.14)	0.75 (0.09)	**0.33 (0.04)**	**4.56 (0.14)**
Once a day or less	194 (67.6)	**2.01 (0.07)**	1.00 (0.81)	0.75 (0.13)	**0.19 (0.03)**	**3.93 (0.18)**
**Tooth brushing**						
<2/day	76 (27.1)	2.17 (0.16)	0.89 (0.15)	0.67 (0.14)	**0.34 (0.05)**	4.03 (0.38)
≥ 2/day	204 (72.9)	2.19 (0.10)	1.01 (0.09)	0.76 (0.09)	**0.18 (0.03)**	4.22 (0.23)
**dmft ≥1**						
Yes	133 (51.4)	**2.36 (0.14)**	0.99 (0.12)	0.89 (0.13)	**0.43 (0.07)**	**4.69 (0.21)**
No	126 (48.7)	**2.00 (0.05)**	1.10 (0.12)	0.84 (0.12)	**0.20 (0.04)**	**3.90 (0.19)**
**dt≥1**						
Yes	45 (18.2)	0.58 (0.13)	0.51 (0.13)	0.36 (0.11)	**0.43 (0.05)**	4.22 (0.54)
No	202 (81.8)	0.70 (0.06)	0.60 (0.06)	0.39 (0.05)	**0.25 (0.04)**	4.33 (0.25)
**Self-rate oral health**						
Ok/poor	116 (39.5)	**2.83 (0.12)**	**1.50 (0.12)**	**1.23 (0.12)**	0.28 (0.05)	**5.73 (0.30)**
Ex/Very good/good	178 (60.5)	**1.85 (0.10)**	**0.73 (0.10)**	**0.47 (0.10)**	0.22 (0.06)	**3.33 (0.24)**

Patterns where expected values (p<0.05)were found are displayed in bold. For example, it was expected that children with worse self-rated oral health would display higher CPQ scores, indicating worse OHRQoL.

^a^1AUS$ = 0.7US$

**Table 8:** Mean (SE) scores for 8-item CPQ and individual items by sample characteristics among children aged 11–13 years.

		The child perception questionnaire (CPQ)				
		Oral symptoms	Functional limitation	Emotional wellbeing	Social wellbeing	CPQ
	N (%)	Mean (SE)	Mean (SE)	Mean (SE)	Mean (SE)	Mean (SE)
Total	461	2.32 (0.07)	1.09 (0.08)	0.55 (0.05)	0.40 (0.05)	4.35 (0.19)
**Sex**						
Boy	232 (50.3)	2.44 (0.10)	1.17 (0.11)	0.51 (0.08)	0.43 (0.06)	4.55 (0.27)
Girl	229 (49.7)	2.19 (0.10)	1.01 (0.11)	0.58 (0.08)	0.37 (0.06)	4.15 (0.26)
**Parent’s Education level**						
High school or less	178 (40.6)	2.33 (0.12)	1.14 (0.12)	**0.59 (0.04)**	0.40 (0.05)	**4.47 (0.12)**
Trade to diploma	106 (24.2)	2.30 (0.15)	0.96 (0.16)	**0.42 (0.05)**	**0.29 (0.03)**	**4.05 (0.09)**
Tertiary	154 (35.2)	2.35 (0.13)	1.06 (0.13)	0.50 (0.07)	**0.44 (0.05)**	4.33 (0.23)
**Household income**						
< ^a^AUS$ 40k	165 (39.9)	2.28 (0.12)	1.15 (0.13)	**0.64 (0.06)**	**0.46 (0.06)**	**4.63 (0.17)**
AUS$ 40-60k	127 (30.7)	2.44 (0.14)	0.92 (0.15)	**0.41 (0.06)**	**0.24 (0.05)**	**4.01 (0.15)**
>AUS$ 60k	122 (29.5)	2.19 (0.14)	1.00 (0.14)	0.52 (0.10)	0.39 (0.08)	4.10 (0.26)
**Soft drink daily**						
Twice a day or more	189 (42.8)	**2.45 (0.06)**	**1.19 (0.07)**	0.53 (0.07)	0.44 (0.06)	**4.59 (0.17)**
Once a day or less	253 (57.2)	**2.17 (0.08)**	**1.00 (0.08)**	0.54 (0.08)	0.36 (0.07)	**4.16 (0.09)**
**Sweet drink daily**						
Twice a day or more	147 (33.3)	2.34 (0.09)	1.09 (0.10)	0.59 (0.10)	**0.56 (0.07)**	**4.99 (0.25)**
Once a day or less	295 (66.7)	2.31 (0.13)	1.07 (0.14)	0.51 (0.08)	**0.33 (0.05)**	**4.00 (0.23)**
**Tooth brushing**						
<2/day	145 (34.1)	**2.58 (0.13)**	1.07 (0.14)	0.54 (0.09)	0.40 (0.08)	**4.65 (0.24)**
≥ 2/day	280 (65.9)	**2.20 (0.05)**	1.09 (0.10)	0.48 (0.06)	0.35 (0.06)	**3.80 (0.19)**
**DMFT ≥1**						
Yes	101 (29.0)	**2.49 (0.12)**	1.15 (0.16)	**0.71 (0.11)**	**0.54 (0.05)**	**4.89 (0.30)**
No	247 (71.0)	**2.10 (0.08)**	1.02 (0.10)	**0.42 (0.08)**	**0.31 (0.07)**	**3.90 (0.20)**
**DT≥1**						
Yes	27 (7.2)	**2.39 (0.09)**	1.07 (0.09)	**0.75 (0.06)**	0.44 (0.19)	4.36 (0.80)
No	350 (92.8)	**2.08 (0.07)**	1.00 (0.32)	**0.49 (0.07)**	0.41 (0.05)	4.34 (0.22)
**Self-rate oral health**						
Fair/poor	39 (12.3)	**3.00 (0.23)**	**2.08 (0.25)**	**1.44 (0.17)**	**0.85 (0.14)**	**7.36 (0.58)**
Ex/Very good/good	278 (87.7)	**2.23 (0.09)**	**0.93 (0.25)**	**0.36 (0.06)**	**0.32 (0.05)**	**3.83 (0.22)**

Patterns where expected values (P<0.05) were found are displayed in bold. For example, it was expected that children with worse self-rated oral health would display higher CPQ scores, indicating worse OHRQo

^a^1AUS$ = 0.7US$

## Discussion

We aimed to develop and validate short-form 4-item CPQ_8-10_ and CPQ_11-14_ instruments for use among school children in Australia. Our findings indicate that the 4-item CPQ_8-10_ and CPQ_11-14_ instruments have adequate validity and acceptable responsiveness. While the reliability of the 4-item CPQ_11-14_ was acceptable for comparisons at a group level, the reliability of the 4-item CPQ_8-10_ should be evaluated in future studies. The 4-item CPQ _8–10_ and CPQ _11–14_ were also unidimensional, indicating that both short forms measure a unique overall dimension of children’s OHRQoL.

The development of the 37-item CPQ_11-14_ constituted the first questionnaire to evaluate OHRQoL among children. The importance of a tailored instrument was that children's cognitions about health, such as their perceptions regarding OHRQoL, are age-dependent, resulting from children's stage of cognitive and language development [11]. Despite its originality and excellent psychometric properties, the response burden associated with answering 37 items, especially for children aged 11 to 14, led researchers to advocate for shorter versions [30]. Over the last two decades, the 16-item and 8-item CPQ_11-14_ [16] and 25-item CPQ_8-10_ [12] were developed and their good psychometric properties were replicated by independent studies [31, 32].

However, the 8- and 16-item CPQ forms have not been included in national and state-wide surveys applied in schools or longitudinal studies because child OHRQoL needs to be evaluated with a multitude of other outcomes, including general health, mental health and educational attainment. Managers of large surveys, as reported previously, have concerns regarding response burden. A meta-analysis conducted by Rolstad et al. [15] demonstrated the effect of questionnaire length on response burden, indicating a greater chance of response when patients were presented with a comparatively shorter questionnaire. Thus, reducing response burden is the rationale driving researchers to investigate the development of questionnaires with a minimum number of items [15].

Addition of child OHRQoL data would not only contribute to the overall richness and comprehensiveness of large, multidisciplinary surveys of child health, development and wellbeing, but provide tangible evidence for health policy translation in terms of the importance of oral health in school productivity, social engagement and quality of life across the life course. The data would yield important information for fair and equitable child dental service provision, and provide a valuable monitoring and surveillance tool in the policy, health and education sectors. There are three main ways, in a research sense, of how capturing oral health-related items in large, population-based surveys would give more power to answer key oral health research questions: (1) samples would be large and representative; (2) collection over time would enable trajectories to be calculated and downstream consequences (for example, experience of dental disease in adulthood) more accurately predicted and; (3) it would be possible to stratify by geographic location or other subgroups of children (for example, socially disadvantaged), which is critical when oral health resources need to be targeted because of resource constraints.

In our study, we evaluated the development of a CPQ version with a minimum number of items, comprising only one item for each of the 4 OHRQoL domains. Our findings showed that the 4-item CPQ had equivalent versions (that is, they should include the same 4 items) for children aged 8 to 10 and aged 11 to 14. These 4 items were chosen based on the highest factor loading on the overall OHRQoL factor, indicating that these items better discriminated the children according to their levels of OHRQoL. For example, item FL_1_ (“Difficulty biting or chewing firm foods”) was chosen over item FL_2_ (“Taken longer than others to eat a meal”) to measure “Functional limitation”. It seems reasonable that item FL_1_ measured “Functional limitation” more accurately since dental diseases, such as tooth decay, often lead to difficulties in chewing food [33]. On the other hand, when a child “Takes longer than others to eat a meal”, this can happen due to other reasons than dental problems, such as time spent watching television or using smartphones [34, 35].

The findings showed that the 4-item CPQ_8-10_ and CPQ_11-14_ are unidimensional measures, meaning the total score should be computed summing all 4 items. That is, the 4 items measure distinct domains of OHRQoL (Oral Symptoms, Functional Limitation, Emotional Wellbeing and Social Wellbeing) but these domains are part of an overall *broader* construct of OHRQoL. Despite the differences between domains, for example between a physiological domain such as Functional Limitation (“Difficulty biting or chewing firm foods”) and a psychological domain such as Emotional wellbeing (“Been upset because of your teeth or mouth”), these 4 domains were all related to broader low quality of life due to oral health problems.

There is one point regarding the 4-item CPQ_8-10_ and CPQ_11-14_ which warrant further investigation. The reliability was below standards for group comparison (>.70) [36] in the children aged 8 to 10 group; while, for children aged 11 to 14, reliability had a bordering but still acceptable value. Reliability is a function of questionnaire length *and* trait variance. Hence, in the event that the 4-item CPQ_8-10_ and CPQ_11-14_ is included in government-funded surveys, these surveys will contain tens of thousands of children, with sample sizes more than ten times bigger than our study sample. With larger sample sizes, the higher sample heterogeneity regarding OHRQoL (i.e. higher trait variance) will possibly improve reliability despite the shortened questionnaire. This possibility, however, needs to be investigated and is a topic for future research. For now, due to the decreased reliability, the application and interpretation of the 4-item CPQ_8-10_ results need to be conducted with caution. It is well-know, for example, that decreased reliability can lead to effect attenuation [37]. For example, diminished reliability can decrease the *estimate* of the OHRQoL effect (as measured by the 4-item CPQ_8-10_ total score) on a chosen outcome (or vice-versa). While this study presented initial good results regarding the 4-item CPQ_8-10_ psychometric properties, future independent studies need to further investigate the instrument’s reliability.

Finally, the 4-item CPQ_8-10_ and CPQ_11-14_ displayed good criterion validity since expected score patterns were found in the majority of groups evaluated. For instance, higher mean scores (indicating worse OHRQoL) were found in children with worse self-rated oral health and higher soft drink consumption among others. Although the observed trend was expected—the higher score was in the lower income groups among children aged 8–10 years—there was no strong evidence demonstrated. One reason could be due to the many missing values (more than 12%).

## Conclusion

This study was the first to propose and evaluate the psychometric properties of the 4-item CPQ_8-10_ and CPQ_11-14_ questionnaire. The upsurge of large governmental surveys that evaluate multiple health outcomes requires short questionnaires. We showed initial evidence that the 4-item CPQ_8-10_ and CPQ_11-14_ questionnaires are unidimensional instruments that can measure OHRQoL in children aged 8 to 10 and aged 11 to 14. The strengths of the study include: (1) it is not only the shortest form of CPQ, but also the only age-appropriate CPQ tool which can be used to assess school children’s OHRQoL and; (2) the development and testing was conducted among a large population of school children, which is especially suitable for longitudinal cohort follow-up. We acknowledge that the 4 item CPQ_11-14_ was better able to capture the oral health of children aged 11–14 years compared to the 4-item CPQ_8-11_ that assesses children aged 8–11 years. We recommend further validation in child groups from other parts of the world.
